# Expression of miR-210, miR-137, and miR-153 in Patients with Acute Cerebral Infarction

**DOI:** 10.1155/2021/4464945

**Published:** 2021-12-02

**Authors:** Hongtao Tian, Yan Zhao, Chao Du, Xiao Zong, Xiuping Zhang, Xia Qiao

**Affiliations:** ^1^Department of Neurosurgery, Qingdao Haizi Medical Group, Qingdao, 266000 Shandong Province, China; ^2^Hemodialysis Room, Qingdao Haizi Medical Group, Qingdao, 266000 Shandong Province, China; ^3^Qingdao Haizi Medical Group, Qingdao, 266000 Shandong Province, China; ^4^Department of Ophthalmology, Liaocheng Guangming Eye Hospital, Liaocheng, 252000 Shandong Province, China; ^5^Department of Neurology, Liaocheng People's Hospital, Liaocheng, 252000 Shandong Province, China

## Abstract

**Aim:**

To explore the expression levels of miR-210, miR-137, and miR-153 in patients with acute cerebral infarction. *Material and Methods*. 76 patients with acute cerebral infarction treated in our hospital from April 2016 to October 2017 were enrolled as the observation group. Another 64 normal patients were selected as the control group. The patients were divided into the death and survival groups based on 1-year mortality of patients. qRT-PCR was used to detect the expression of miR-210, miR-137, and miR-153 in the serum of each group. Receiver operating characteristic (ROC) curve was employed to analyze the diagnostic value and predictive value of miR-210, miR-137 and miR-153 death in patients. The correlation between miR-210, miR-137, and miR-153 in the serum of the observation group was analyzed by Pearson's test.

**Results:**

Levels of miR-210 and miR-137 in the observation group were significantly lower than those in the control group, while levels of miR-153 in the observation group were significantly higher than those in the control group (all *P* < 0.05). The ROC curve of diagnosis of acute cerebral infarction showed that the area under curve of miR-210 was 0.836, that of miR-137 was 0.843, and that of miR-153 was 0.842. The 1-year survival rate was 71.05%. The 1-year survival of the low-expression group of miR-210 and miR-137 was significantly lower than that of the high-expression group, while the 1-year survival of the low-expression group of miR-153 was significantly higher than that of the high-expression group (all *P* < 0.05). The ROC curve for predicting death showed that the area under curve of miR-210 was 0.786, that of miR-137 was 0.824, and that of miR-153 was 0.858. Pearson's correlation analysis showed that the expression of miR-210 was positively correlated with that of miR-137, while miR-137 was negatively correlated with that of miR-153 and miR-210 was negatively correlated with that of miR-153.

**Conclusion:**

miR-210, miR-137, and miR-153 have a certain value in the diagnosis and prediction of 1-year death of acute cerebral infarction and may be potential diagnostic and predictive indicators.

## 1. Introduction

Cerebral infarction is a kind of brain injury caused by obstruction of blood supply in the brain. The patients usually have sudden onset and will show symptoms in a short time. The incidence and mortality of cerebral infarction are much higher than those of other brain injury diseases [1, 2]. And most of acute stroke is acute cerebral infarction, which has become the main cause of global disability events [3, 4]. With the development of social aging, its incidence shows an upward trend [5]. The number of cerebral infarction patients worldwide was 33 million in 2010, and it would increase to 77 million by 2030 according to epidemiological speculation [6]. Therefore, we need some indicators to diagnose the disease and predict the prognosis, so that medical staff can carry out targeted and effective treatment according to the predicted situation.

MicroRNA is a class of small-molecule noncoding short-stranded RNA that regulates and influences the occurrence and development of diseases such as cancer and cardiovascular and cerebrovascular diseases by their target proteins [7–9]. However, miR-210 can regulate brain-derived neurotrophic factor (BDNF). When miR-210 is overexpressed, microvessel density and the number of neuronal progenitor cells in the brain of ischemic mice can be increased, thus improving the neurobehaviour of ischemic mice [10]. The research progress of the role of BDNF in neural plasticity, neural protection, and neurogenesis may provide important information for the formulation of new poststroke rehabilitation strategies. It plays a regulatory role in poststroke kinematic learning and rehabilitation. When stroke patients recover, their BDNF will rise and protect the nerve [11–13]. Other miRNAs also regulate BDNF and may play a regulation role in stroke situations. miR-137 is associated with schizophrenia and some neurological disorders. Studies in [14] have suggested that miR-137 regulates the signal pathways related to schizophrenia and the convergence mechanism regulates neuronal responses to Nrg1*α* and BDNF, so as to alter the neural development, leading to the risk of schizophrenia. miR-153 is closely related to autism. High expression of miR-153 can inhibit the activation of the JAK-STAT signaling pathway by LEPR, thereby enhancing the expression of BDNF and the proliferation of hippocampal neurons and improving the condition of autistic mice [15]. miR-210, miR-137, and miR-153 all have the effect of regulating BDNF, and BDNF also plays a regulatory role in the development of cerebral infarction. However, the clinical effects of the expressions of miR-210, miR-137 and miR-153 in patients with acute cerebral infarction are still unclear.

Therefore, this study explored the clinical value of miR-210, miR-137, and miR-153 in patients with acute cerebral infarction and provided a reference for clinical treatment.

## 2. Method and Data

### 2.1. Clinical Data of Patients

76 patients with acute cerebral infarction treated in our hospital from April 2016 to October 2017 were selected as the observation group in this study, including 45 males and 31 females, with an average age of 57.0 ± 6.4 years. Another 64 patients with normal physical examination were collected as the control group, including 42 males and 22 females, with an average age of 56.4 ± 6.2 years. The study was conducted with the approval of the Medical Ethics Committee. All patients were informed and signed the informed consent.

### 2.2. Inclusion of Exclusion Criteria

#### 2.2.1. Inclusion Criteria

Acute stroke was diagnosed on the basis of imaging and pathology. The diagnostic criteria were in accordance with the guidelines issued by the American Heart Association Stroke Committee in 2013 [16]. All patients were hospitalized within 6 hours after onset of the disease. The patients could be followed up by telephone with completed clinical data.

#### 2.2.2. Exclusion Criteria

The exclusion criteria are the following: patients with severe liver and kidney dysfunction, patients with malignant tumor history, patients who complicated with other malignant tumors, patients with severe cardiovascular and cerebrovascular diseases, patients with severe inflammation, and pregnant or lactating women.

### 2.3. Sample Collection

Five milliliters of venous blood was collected from health examinees in the morning and another five milliliters from patients in observation group after admission. The venous blood in the procoagulation tube was centrifuged at 24°C for 10 minutes at the speed of 3000 rpm. The serum was collected for the PCR test and stored at -80°C.

### 2.4. Major Kits and Instruments

The following are used in the study: hematology analyzer (Siemens, Germany, ADVIA2120i); PCR (ABI Company, USA, 7500); total RNA extraction kit EasyPure microNA Kit and reverse transcription + PCR kit TransScript microNA First-Strand cDNA Synthesis SuperMix (TransGen Biotech Company, Beijing, China, ER601-01, AT351-01); and primers (Shanghai Shenzhen University of Technology). The primers were designed and synthesized by Shanghai Biotechnology Co., Ltd. as shown in Table 1.

### 2.5. PCR Detection Method

The EasyPure miRNA Kit was used to extract the total RNA from serum, and the total RNA after extraction was tested for its purity, concentration, and integrity by ultraviolet spectrophotometer and agarose gel electrophoresis. Reverse transcription with total RNA using TransScript® miRNA RT Enzyme Mix and 2 × TS miRNA Reaction Mix was operated in strict accordance with the manufacturer's kit. Subsequently, PCR amplification experiments were carried out. The system of PCR reaction was as follows: 1 *μ*L of cDNA, 0.4 *μ*L of upstream and downstream primers, 10 *μ*L of 2 × TransTaq® Tip Green qPCR SuperMix, 0.4 *μ*L of Passive Reference Dye (50x), and finally ddH_2_O added to 20 *μ*L. The conditions of PCR reaction were as follows: predenaturation at 94°C for 30 s, denaturation at 94°C for 5 s, annealing at 60°C for 30 s, and a total of 40 cycles were performed. Each sample had three repetitive holes, and the experiment was carried out three times. In this study, U6 was taken as an internal reference and 2^-△ct^ was used to analyze the data.

### 2.6. Follow-Up

A total of 76 patients or their families were followed up by telephone and visited every two months, lasting for one year.

### 2.7. Observation Indicators

#### 2.7.1. Main Outcome Measure

The levels of miR-210, miR-137, and miR-153 were compared between the observation group and the control group. And 1-year survival of the patients was counted. Then, the receiver ROC was used to analyze the diagnostic value of miR-210, miR-137, and miR-153 in patients with acute cerebral infarction and predictive value of one-year mortality.

#### 2.7.2. Secondary Outcome Measures

The secondary outcome measures following are follows: clinical data of the two groups; miR-210, miR-137, and miR-153 levels in survival patients and death patients; and correlation analysis between miR-210, miR-137, and miR-153 in the observation group.

### 2.8. Statistical Analysis

This study used SPSS20.0, a medical statistical analysis software (Chicago SPSS Co., Ltd.), to analyze the collected data. And GraphPad Prism 7 (San Diego GraphPad Software Co., Ltd.) was used to draw pictures of the collected data. A chi-square test was used for counting data utilization (%), represented by *X*2. Measurement data were expressed by the means ± standard deviation (mean ± SD), which were in a normal distribution. The independent sample *t*-test was used to compare the two groups, expressed by *t*. ROC was used to evaluate the diagnostic value of miR-210, miR-137, and miR-153 in patients with acute cerebral infarction and the predictive value of 1-year mortality. K-M survival analysis revealed one-year survival condition of patients and analyzed by a log rank test. Pearson's test was used to analyze the correlation between miR-210, miR-137, and miR-153 in patients. *P* < 0.05 was considered statistically significant.

## 3. Results

### 3.1. Clinical Data of Patients

Clinical data of two groups were collected to compare. The results showed that there were no significant differences in gender, age, BMI, past medical history (hypertension, diabetes, hyperlipidemia), smoking history, alcoholism history, residence, platelet count, total cholesterol, and triglyceride between the two groups (all *P* > 0.05), as shown in Table 2.

### 3.2. Expression of miR-210, miR-137, and miR-153 in Two Groups of Patients

By comparing the expression of miR-210, miR-137, and miR-153, we found that miR-210 in the observation group (1.18 ± 0.26) was significantly lower than that in the control group (1.64 ± 0.48) (*P* < 0.05), and miR-137 in the observation group (0.84 ± 0.24) was significantly lower than that in the control group (1.26 ± 0.31) (*P* < 0.05), but miR-153 in the observation group (1.52 ± 0.45) was significantly higher than that in the control group (0.96 ± 0.36) (*P* < 0.05) (see Figure 1).

### 3.3. Diagnostic Value of miR-210, miR-137, and miR-153 in Patients with Acute Cerebral Infarction

The diagnostic value of ROC analysis in patients with acute cerebral infarction was drawn by analyzing the expression of miR-210, miR-137, and miR-153 in the observation group and the control group. The area under curve of miR-210 was 0.836 (95% CI: 0.764-0.907); the area under curve of miR-137 was 0.843 (95% CI: 0.776-0.909); and the area under curve of miR-153 was 0.842 (95% CI: 0.778-0.906) (see Figure 2 and Table 3).

### 3.4. One-Year Survival in the Two Groups

According to the one-year survival statistics of the patients in the observation group, 76 patients were followed up, and 0 patient failed to be followed up. 22 patients died, and 54 patients survived within one year, with a survival rate of 71.05%. The patients were divided into the high and low-expression groups based on the median expression of miR-210, miR-137, and miR-153. The K-M curve showed that the one-year survival of miR-210 and miR-137 in the low-expression group was significantly lower than that in the high-expression group (*P* < 0.05) and the one-year survival of miR-153 in the low-expression group was significantly higher than that in the high-expression group (*P* < 0.05, see Figure 3).

### 3.5. Expression of miR-210, miR-137, and miR-153 in the Survival and Death Groups of Patients

According to the one-year survival condition of the patients in the observation group, the patients were divided into the survival group and the death group. After comparing the expressions of miR-210, miR-137, and miR-153 in the two groups, it was found that miR-210 (1.01 ± 0.13) in the death group was significantly lower than that in the survival group (1.26 ± 0.20) (*P* < 0.05) and miR-137 (0.65 ± 0.15) in the death group was significantly lower than that in the survival group (0.94 ± 0.21) (*P* < 0.05). miR-153 in the death group (1.84 ± 0.23) was significantly higher than that in the survival group (1.39 ± 0.38) (*P* < 0.05, see Figure 4).

### 3.6. Predictive Value of miR-210, miR-137, and miR-153 in Patients with 1-Year Mortality

The predictive value of ROC analysis in patients with one-year mortality was drawn by analyzing the expression of miR-210, miR-137, and miR-153 in the survival and death groups. It was found that the area under curve of miR-210 was 0.786 (95% CI: 0.680-0.893); the area under curve of miR-137 was 0.824 (95% CI: 0.730-0.918); and the area under curve of miR-153 was 0.858 (95% CI:0.771-0.945) (see Figure 5 and Table 4).

### 3.7. Correlation Analysis between miR-210, miR-137, and miR-153 in the Observation Group

Through Pearson's analysis of the relationship between miR-210, miR-137, and miR-153 in the observation group, it was found that the expression of miR-210 was positively correlated with miR-137, while the expression of miR-137 was negatively correlated with miR-153, and the expression of miR-210 was negatively correlated with miR-153, as shown in Figure 6.

## 4. Discussion

Acute cerebral infarction can cause severe brain damage [17, 18]. Some of the microRNAs that are proposed to be expressed in the brain will also change. Some of these microRNAs will also change with the severity and alleviation of the disease. And some of them are expected to serve as potential diagnostic and predictive indicators of disease or as a new direction of treatment [19, 20].

MicroRNA-210, a master and pleiotropic hypoxia-miRNA, plays multiple roles in brain ischemia. The current finding that pretreatment with miR-210 inhibitor significantly attenuated hypoxia-ischemia- (HI-) induced brain infarct size suggests that miR-210 has a functional significance in the pathophysiology of HI-induced brain injury in the developing brain. This finding is consistent with the previous study, which found that silencing miR-210 with miR-210-LNA via intracerebroventricular or intranasal delivery induced a neuroprotective effect on neonatal brain HI insult [21]. Wang et al. [22] provide new evidence that miR-210 may be involved in the nicotine-induced epigenetic mechanism. Perinatal nicotine exposure enhances miR-210 expression, but decreases the neurotrophic protein (BDNF/TrkB) expression in neonatal brains and subsequent development of brain hypoxic-ischemia sensitive phenotype in neonates. Thomas et al. reported that miR-137 regulates target proteins within the phosphoinositide 3-kinase-Akt-mechanistic target of rapamycin (PI3K-Akt-mTOR) pathway, which acts downstream of ErbB receptors. Nrg1*α* increases phospho-S6 (Ser235/236) levels, mRNA translation, AMPA receptor levels, and outgrowth in the dendrites of primary neurons. Chronic inhibition of miR-137 reverses or abolishes the effects of Nrg1*α* signaling by all measures. Inhibition of miR-137 also abolishes dendritic outgrowth and mRNA translation induced by BDNF [14]. miR-153, an intronic miRNA recognized as a modulator of alpha-synuclein at posttranscription level, has been identified to be a significant component of the brain with an example that reflects synuclein expression in different tissues in the period of neuronal development, indicating that they take coordinated effects in alpha-synuclein. As You et al. described [15], miR-153 blocked the JAK-STAT signaling pathway through the inhibition of leptin receptor (LEPR), thus regulating BDNF expression and proliferation of hippocampal neurons. Fragkouli and Doxakis also suggested that miR-153 provides protection for neurons against death by downregulating the mTOR signaling pathway [23].

In this study, the expression of miR-210, miR-137, and miR-153 in the observation group and the control group were detected by PCR. The results showed that the expression of miR-210 and miR-137 in the observation group was significantly lower than that in the control group, while the expression of miR-153 was significantly higher than that in the control group. In the study of Jiang et al. [24], it was mentioned that vagus nerve stimulation can exert neuroprotective effects on cerebral ischemia rats, which thus increased expression of miR-210 and decreased antioxidative stress response. The benefits of VNS are weakened after miR-210 knockdown, so they believe that miR-210 mediates antioxidant stress to improve cerebral ischemia. Other studies have also shown that the expression of miR-137 in astrocytes from the hypoxic and glucose-deficient environment to normal environment will also increase [25]. Therefore, we suspect that the expression of miR-210 and miR-137 may decrease with the alleviation of the patient's condition. At the same time, the difference between the two groups also suggests that miR-210, miR-137, and miR-153 may have a potential diagnostic value in acute cerebral infarction. Therefore, we used the ROC curve to find that the area under curve of miR-210 is 0.836. When the cut-off point is 1.401, the best specificity and sensitivity are 81.58% and 71.88%. The area under curve of miR-137 is 0.843. When the cut-off point is 1.121, the best specificity and sensitivity are 70.31% and 55.84%. The area under curve of miR-153 is 0.842. When the cut-off point is 1.299, the best specificity and sensitivity are 73.68% and 81.25%. These results suggest that miR-210, miR-137, and miR-153 may be potential diagnostic indicators for acute cerebral infarction. Yang et al. [26] also compared the expression of miR-153 in cerebral infarction patients and normal people in their study. It was found that the expression of miR-153 in patients with cerebral infarction was also higher than that in normal people. Then, they also found that miR-153 had a good diagnostic ability in the diagnosis of cerebral infarction through ROC curve analysis, which further confirmed our conclusion.

Death has always been a major threat to acute cerebral infarction. Several studies have found that the severity of admission symptoms, insular infarction, and cerebral infarction in patients with acute cerebral infarction are independent predictors of clinical prognosis [27, 28]. We followed up the patients in the observation group for one year and found that the one-year survival rate was 71.05%. The one-year survival of the low-expression group of miR-210 and miR-137 was significantly lower than that of the high-expression group, while the one-year survival of the low-expression group of miR-153 was significantly higher than that of the high-expression group. The results suggest that the expression of miR-210, miR-137, and miR-153 may predict one-year survival of patients. Therefore, we first compared the expression of miR-210, miR-137, and miR-153 between the death and the survival patients. We found that the expression of miR-210 and miR-137 in the death group was significantly lower than that in the survival group, and the expression of miR-153 was significantly higher than that in the survival group. We then mapped the ROC curves of miR-210, miR-137, and miR-153 predicting death within 1 year based on the expression of survival patients and death patients. We found that the area under curve of miR-210 was 0.786. The optimal specificity and sensitivity were 6.81% and 77.78%, and the area under curve of miR-137 was 0.824. When the cut-off point was 0.867, the best specificity and sensitivity were 85.53% and 95.45%. The area under curve of miR-153 is 0.858. When the cut-off point is 1.609, the best specificity and sensitivity are 81.82% and 75.93%. Therefore, miR-210, miR-137, and miR-153 have a certain predictive value for one-year survival of patients and may become potential predictors.

At the end of the study, we analyzed the relationship between miR-210, miR-137, and miR-153 by Pearson's correlation. It was found that the expression of miR-210 was positively correlated with miR-137, miR-137 was negatively correlated with miR-153, and miR-210 was negatively correlated with miR-153, suggesting that there may be a close relationship between miR-210, miR-137, and miR-153. However, there are still some limitations in this study. Firstly, our study did not include the corresponding treatment research. Whether the indicators before and after the study will change is not clear. Secondly, this study did not collect the expression of miR-210, miR-137, and miR-153 in patients after being discharged from hospital. Finally, this study was only used as a clinical trial. It is not clear what the relationship between miR-17-5p and NLR is. Therefore, we hope to add some basic experiments in future research to explore the relationship between miR-17-5p and NLR and to verify the results of our research.

In summary, miR-210, miR-137, and miR-153 have a certain value in the diagnosis and prediction of 1-year death of acute cerebral infarction and may be potential diagnostic and predictive indicators.

## Figures and Tables

**Figure 1:** Expression of miR-210, miR-137 and miR-153 in the two groups. (a) Expression of miR-210 in the observation group was significantly lower than that in the control group (*t* = 7.197, *P* < 0.001). (b) miR-137 in the observation group was significantly lower than that in the control group (*t* = 9.029, *P* < 0.001). (c) miR-153 in the observation group was significantly higher than that in the control group (*t* = 8.024, *P* < 0.001). ∗∗∗ indicates *P* < 0.001.

**Figure 2:** ROC of miR-210, miR-137 and miR-153 in the diagnosis of acute cerebral infarction. The area under curve of miR-210 is 0.836 (95% CI: 0.764-0.907), the area under curve of miR-137 is 0.843 (95% CI: 0.776-0.909), and area under curve of miR-153 is 0.842 (95% CI: 0.778-0.906).

**Figure 3:** (a) The survival of miR-210 in the low-expression group was significantly lower than that of the high-expression group (*P* = 0.017). (b) The survival of miR-137 in the low-expression group was significantly lower than that of the high-expression group (*P* = 0.043). (c) The survival of miR-153 in the low-expression group was significantly higher than that of the high-expression group (*P* = 0.002).

**Figure 4:** Expression of miR-210, miR-137, and miR-153 in survival and death patients. (a) miR-210 in the death group was significantly lower than that in the survival group (*t* = 5.405, *P* < 0.001). (b) miR-137 in the death group was significantly lower than that in the survival group (*t* = 5.884, *P* < 0.001). (c) miR-153 in the death group was significantly higher than that in the survival group (*t* = 5.170, *P* < 0.001). ∗∗∗ indicates *P* < 0.001.

**Figure 5:** ROC of miR-210, miR-137, and miR-153 predicted patient death. The area under curve of miR-210 was 0.786 (95% CI: 0.680-0.893), the area under curve of miR-137 was 0.824 (95% CI: 0.730-0.918), and area under curve of miR-153 was 0.858 (95% CI: 0.771-0.945).

**Figure 6:** Correlation between miR-210, miR-137, and miR-153 in the observation group. (a) Expression of miR-210 was positively correlated with miR-137 (*r* = −0.705, *P* < 0.001). (b) Expression of miR-137 was negatively correlated with miR-153 (*r* = −0.620, *P* < 0.001). (c) Expression of miR-210 was negatively correlated with miR-153 (*r* = 0.659, *P* < 0.001).

**Table 1:** Primer sequences.

Gene	Upstream primer	Downstream primer
miR-210	5′-GTGCAGGGTCCGAGGT-3′	5′-TATCTGTGCGTGTGACAGCGGCT-3′
miR-137	5′-GAAATCCGACAGCTTAAGGAGGTTTGA-3′	5′-CATTGCACAGATAGGATTTGATTTACT-3′
miR-153	5′-UUGCAUAGUCACAAAAGUGAUC-3′	5′-TCCACCACCCAGTTGCTGTA -3′
U6	5′-CTCGCTTCGGCAGCACA-3′	5′-AACGCTTCACGAATTTGCGT-3′

**Table 2:** Clinical data of patients.

Factors	Observation group (*n* = 76)	Control group (*n* = 64)	*t*/*χ*^2^/*Z* value	*P* value
Gender				
Male	45 (59.21)	42 (65.63)	0.608	0.436
Female	31 (40.79)	22 (34.38)		
Age	57.0 ± 6.4	56.4 ± 6.2	0.561	0.576
BMI (kg/m^2^)	23.65 ± 1.82	24.04 ± 1.97	1.216	0.226
Past medical history				
Hypertension	19 (25.00)	21 (32.81)	1.039	0.308
Diabetes	13 (17.11)	10 (15.63)	0.055	0.814
Hyperlipidemia	8 (10.53)	8 (12.50)	0.134	0.715
History of smoking				
Yes	19 (25.00)	18 (28.13)	0.175	0.676
No	57 (75.00)	46 (71.88)		
History of alcohol abuse				
Yes	9 (11.84)	10 (15.63)	0.424	0.515
No	67 (88.16)	54 (84.38)		
Place of residence				
City	58 (76.32)	50 (78.13)	0.065	0.800
Rural	18 (23.68)	14 (21.88)		
Platelet count (×10^9^/L)	152.93 ± 54.41	147.23 ± 51.62	0.632	0.528
Total cholesterol (mmol/L)	6.58 ± 0.87	6.54 ± 0.83	0.782	0.277
Triglyceride (mmol/L)	3.32 ± 0.74	3.47 ± 0.81	1.144	0.255
Location of infarction				
Frontal lobe	12 (15.79)			
Temporal lobe	10 (13.16)			
Parietal lobe	9 (11.84)			
Occipital lobe	9 (11.84)			
Basal ganglia	10 (13.16)			
Thalamus	11 (14.47)			
Cerebellum	10 (13.16)			
Brainstem	5 (6.58)			
Infarct size				
Lacunar infarction	39 (51.32)			
Medium area infarction	23 (30.26)			
Massive infarction	14 (18.42)			

**Table 3:** ROC curve data.

Indicators	AUC	95% CI	Specificity	Sensitivity	Youden index	Cut-off
miR-210	0.836	0.764~0.907	81.58%	71.88%	53.46%	1.401
miR-137	0.843	0.776~0.909	85.53%	70.31%	55.84%	1.121
miR-153	0.842	0.778~0.906	73.68%	81.25%	54.93%	1.299

AUC: area under curve; cut-off: cut point.

**Table 4:** ROC curve data.

Indicators	AUC	95% CI	Specificity	Sensitivity	Youden index	Cut-off
miR-210	0.786	0.680-0.893	68.18%	77.78%	45.96%	1.115
miR-137	0.824	0.730-0.918	85.53%	95.45%	80.98%	0.867
miR-153	0.858	0.771-0.945	81.82%	75.93%	57.75%	1.609

AUC: area under curve; cut-off: cut point.

## Data Availability

The datasets used and/or analyzed during the current study are available from the corresponding author on reasonable request.
